# Sarcosine Up-Regulates Expression of Genes Involved in Cell Cycle Progression of Metastatic Models of Prostate Cancer

**DOI:** 10.1371/journal.pone.0165830

**Published:** 2016-11-08

**Authors:** Zbynek Heger, Miguel Angel Merlos Rodrigo, Petr Michalek, Hana Polanska, Michal Masarik, Vitezslav Vit, Mariana Plevova, Dalibor Pacik, Tomas Eckschlager, Marie Stiborova, Vojtech Adam

**Affiliations:** 1 Department of Chemistry and Biochemistry, Mendel University in Brno, Zemedelska 1, CZ-613 00, Brno, Czech Republic; 2 Central European Institute of Technology, Brno University of Technology, Purkynova 123, Brno, CZ-612 00, Czech Republic; 3 Department of Physiology, Faculty of Medicine, Masaryk University, Kamenice 5, Brno, CZ-625 00, Czech Republic; 4 Department of Urology, University Hospital Brno, Jihlavska 20, Brno, CZ-625 00, Czech Republic; 5 Department of Paediatric Haematology and Oncology, 2nd Faculty of Medicine, Charles University, and University Hospital Motol, V Uvalu 84, CZ-150 06, Prague 5, Czech Republic; 6 Department of Biochemistry, Faculty of Science, Charles University, Albertov 2030, CZ-128 40, Prague 2, Czech Republic; University of Kentucky College of Medicine, UNITED STATES

## Abstract

The effects of sarcosine on the processes driving prostate cancer (PCa) development remain still unclear. Herein, we show that a supplementation of metastatic PCa cells (androgen independent PC-3 and androgen dependent LNCaP) with sarcosine stimulates cells proliferation *in vitro*. Similar stimulatory effects were observed also in PCa murine xenografts, in which sarcosine treatment induced a tumor growth and significantly reduced weight of treated mice (*p* < 0.05). Determination of sarcosine metabolism-related amino acids and enzymes within tumor mass revealed significantly increased glycine, serine and sarcosine concentrations after treatment accompanied with the increased amount of sarcosine dehydrogenase. In both tumor types, dimethylglycine and glycine-*N*-methyltransferase were affected slightly, only. To identify the effects of sarcosine treatment on the expression of genes involved in any aspect of cancer development, we further investigated expression profiles of excised tumors using cDNA electrochemical microarray followed by validation using the semi-quantitative PCR. We found 25 differentially expressed genes in PC-3, 32 in LNCaP tumors and 18 overlapping genes. Bioinformatical processing revealed strong sarcosine-related induction of genes involved particularly in a cell cycle progression. Our exploratory study demonstrates that sarcosine stimulates PCa metastatic cells irrespectively of androgen dependence. Overall, the obtained data provides valuable information towards understanding the role of sarcosine in PCa progression and adds another piece of puzzle into a picture of sarcosine oncometabolic potential.

## Introduction

Sarcosine, also known as *N*-methylglycine, is a non-proteinogenic imino acid occurring as an intermediate and byproduct in glycine synthesis and degradation [1]. In 2009, Sreekumar *et al*. delineated its potential role as urinary, non-invasive biomarker exploitable for early diagnosis of prostate cancer (PCa) [2]. This publication triggered sarcosine research, which resulted in a number of reports studying the connection between this low molecular mass metabolite and PCa diagnostics. Anyway, it has to be noted that the presented results have been somehow contradictory, whereas some of them have demonstrated a positive linkage only [3–5], while some of them have been negative [6, 7]. Thus, the further research is necessary to elucidate the role of sarcosine and its impact on properties of PCa cells.

In our initial study, we revealed that sarcosine supplementation increases the cell migration and decreases the doubling time of malignant prostatic cells *in vitro* [8]. Similar efforts were put by Sudhakaran and colleagues, who described that sarcosine modulates angiogenesis in endothelial cells *in vitro* through PI3K/Akt/mTOR pathway [9]. Moreover, Khan *et al*. demonstrated that sarcosine induces invasion and intravasation in *in vivo* PCa model [10]. Taken together, above mentioned studies showed sarcosine as an oncometabolite and substantiated its role in PCa progression. Although a relatively complex pool of data has been provided, to the best of our knowledge, there still exists a lack of reports on the sarcosine regulatory effects on expression of pivotal genes involved in a cell cycle and apoptosis, which lie beneath the complexity and idiopathy of each cancer [11].

To unravel the putative mechanisms involved in abnormal growth of cancer cells is a complex and vast task requiring powerful tools. One of them is a microarray technology, which accelerated the completion of the human genome project and eliminated numerous previous boundaries [12]. DNA microarrays, also called "gene chips" enable studying of differential gene expression using complex population of RNA [13]. As a result, microarrays provide large gene expression data sets for consequent data mining, which can be carried out using a number of available software applications.

Hence, in our study, we have employed a special type of DNA microarray, based on redox enzyme mediated analysis of cDNA hybridization, to give another piece to the puzzle of sarcosine oncometabolic potential. Using preclinical *in vivo* murine models (PC-3 and LNCaP xenografts); we focused on an investigation of effects of sarcosine treatment on expression of genes involved particularly in a cell cycle and apoptosis. Overall, this study reveals that sarcosine significantly up-regulates the expression of some of those genes, irrespective of androgen dependence status.

## Material and Methods

### Chemicals

Sarcosine standard and other chemicals were purchased from Sigma-Aldrich (St. Louis, MO, USA) in ACS purity, unless noted otherwise.

### Cells

The PC-3 cell line, established from a grade IV androgen-independent prostatic adenocarcinoma and the LNCaP cell line, derived from the left supraclavicular androgen-dependent lymph node PCa metastasis were purchased from the Health Protection Agency Culture Collection (Salisbury, UK). The PC-3 cells were grown in Ham’s F12 medium with 7% foetal bovine serum. The LNCaP cells were grown in RPMI-1640 with 10% fetal bovine serum. Media were supplemented with penicillin (100 U/mL) and streptomycin (0.1 mg/mL). The cells were maintained at 37°C in a humidified incubator with 5% CO_2_. The treatments with sarcosine were initiated after cells reached ~70–80% confluency. Cells were then harvested and washed four times with phosphate-buffered saline (PBS, pH 7.4).

### Viability (MTT) assay

The suspension of 10 000 cells was added to each well of standard microtiter plates. After addition of medium (200 μL), plates were incubated for 2 days at 37°C to ensure cell growth. To determine the effects on cell viability sarcosine in concentrations 0–10 μM was applied. Plates were incubated for 24 h; then, media were removed and replaced by fresh ones, three times a day. Further, for each plate, a medium was replaced by 200 μL of fresh medium containing 50 μL of MTT (5 mg/mL in PBS) and incubated in a humidified atmosphere for 4 h at 37°C, wrapped in aluminum foil. After the incubation, MTT-containing medium was replaced by 200 μL of 99.9% dimethyl sulphoxide (*v*/*v*) to dissolve MTT-formazan crystals. Then, 25 μL of glycine buffer (pH 10.5) was added to all wells and absorbance at 570 nm was immediately determined using the Infinite 200PRO reader (Tecan, Männedorf, Switzerland).

### Light microscopy

For light microscopy, the cells (1×10^5^ at time point 0 h) were cultivated directly on glass microscopy slides (75×25 mm, thickness 1 mm) in medium without and with 1 μM sarcosine. Prior microscopic examination, slides with a monolayer of cells were removed from Petri dishes, rinsed with a medium and PBS and directly used for investigation of their density under an inverted microscope (Olympus IX 71S8F-3, Olympus, Tokyo, Japan).

### Prostate tumor xenograft models and the treatment protocol

Twelve five-week-old male nude athymic BALB/c nu/nu mice were used for xenograft studies. PC-3 or LNCaP cells (5×10^6^) were resuspended in 100 μL of PBS with 20% Matrigel (*v*/*v*, BD Biosciences, Franklin Lakes, NJ, USA) and were then implanted subcutaneously (*s*.*c*.) into the left flank regions of the mice (six mice for PC-3 tumors and six mice for LNCaP tumors) under general anesthesia (1% Narkamon + 2% Rometar, 0.5 mL/100 g of weight). Six mice were utilized as the non-treated controls. All animals were housed in individually ventilated cages at a 12/12 h light/dark cycle and were provided *ad libitum* with standard diet and water. A tumor volume was measured twice per week following the equation (length × width^2^ × 0.5) as well as well-being of the mice. The treatment of mice was carried out *i*.*p*. two times a week for 21 days (total 6 applications) using 100 μL of 5 μM sarcosine solution. After termination by isoflurane inhalation, tumors were excised immediately and stored in RNA*later* (Thermo Fisher, Waltham, MA, USA) prior to further experiments. The use of the animals followed the European Community Guidelines as accepted principles for the use of experimental animals. The experiments were performed with the approval of the Ethics Commission at the Faculty of Medicine, Masaryk University, Brno, Czech Republic.

### Histological procedures

The samples were fixed in formaldehyde (10% *v*/*v*) overnight, subsequently dehydrated in serial ethanol concentrations and embedded in paraffin. Sections were cut at 5 μm, mounted on glass slides, deparaffinized and stained with hematoxylin-eosin (H&E). The microscopic observations were conducted using an Olympus IX 71S8F-3 (Olympus, Tokyo, Japan).

### Ion-exchange chromatography (IEC)

Amino acids (glycine, serine and dimethylglycine) and sarcosine in tumor tissue were determined using IEC with Vis detection after post-column derivatization with ninhydrin (AAA-400, Ingos, Prague, Czech Republic), following conditions employed in our previous study [14].

### Quantitation of glycine-*N*-methyltransferase (GNMT) and sarcosine dehydrogenase (SARDH)

Amounts of GNMT and SARDH in sarcosine treated and non-treated tumors were quantified by human sandwich ELISA kits with HRP-conjugated secondary antibody and 3,3',5,5'-tetramethylbenzidine (TMB) as a substrate (LSBio, Seattle, WA, USA). Color intensity at 495 nm was read in a VersaMax microplate reader (Molecular Devices, Sunnyvale, CA, USA).

### Isolation of RNA and reverse transcription (RT)

High pure total-RNA isolation kit (Roche, Basel, Switzerland) was used for an isolation of tissue RNA. The medium was removed and samples were twice washed with 5 mL of ice-cold PBS. Cells were scraped off, transferred to clean tubes and centrifuged at 20 800×*g* for 5 min at 4°C. After that, lysis buffer was added and RNA isolation was carried out according to manufacturer's instructions. Isolated RNA was used for cDNA synthesis. RNA (500 ng) was transcribed using transcriptor first strand cDNA synthesis kit (Roche) according to manufacturer's instructions. Prepared cDNA (20 μL) was diluted with RNase-free water to a total volume of 100 μL and 5 μL of this solution was employed for microarray analyses.

### Electrochemical microarray

cDNA was biotinylated on its 3’ end using the Biotin 3’ End DNA Labeling Kit (Thermo Scientific, Waltham, MA, USA) following the manufacturer’s instructions. The microarray was performed as previously described by Roth *et al*. [15]. For hybridization, Human Cancer 3711 ElectraSense medium density 4×2k array slides with 1,609 DNA probes (Custom Array, Bothell, WA, USA), were firstly pre-hybridized for 30 min at 50°C using 6× SSPE (0.9 M NaCl, 60 mM sodium phosphate, 6 mM EDTA), 5× Denhardt´s solution and sonicated salmon sperm DNA (100 μg/mL). Then, hybridization of biotin-labeled cDNA was performed at 50°C for 18 h in 6× SSPE and salmon sperm DNA (100 μg/mL). Array chips were rinsed with low ionic strength 3× SSPET (3× SSPE, 0.05% Tween-20) and PBST (2× phosphate-buffered saline, pH 7.4, 0.1% Tween-20) to remove weakly bound DNA. Subsequently, array chips were blocked with biotin blocking solution for 15 min. Chips were then incubated for 30 min with poly-horseradish peroxidase-streptavidin (1:1,000 in PBS containing 1% bovine serum albumin and 0.05% Tween-20). Next, chips were rinsed three times with biotin wash solution and TMB rinse solution, followed by incubation with TMB substrate. Measurements were performed using the ElectraSense detection kit (Custom Array). All post-hybridization processing steps were performed at 25°C.

### Semi-quantitative RT-PCR for validation of selected genes

To confirm selected microarray results we separately performed semi-quantitative RT-PCR (SQ-RT-PCR) of genes with the expression 2.5-fold stronger than non-treated individuals. To adjust the amount of transcribed cDNA, *β-actin* was selected as an internal control. The primer sequences were as follows: 5´-TCCATCGTCCACAGAAAG-3´ (forward) and 5´-AAATGTCCTCCGCAAGCT-3´ (reverse). For designing the primers of tested genes, the sequence information was collected from the NCBI GenBank (www.ncbi.nih.gov). Information about the PCR primers is available upon request to the corresponding author. SQ-RT-PCR experiments were performed in conditions described in our previous study [16]. For evaluation of differences in gene expression between sarcosine treatment and non-treated controls, 10 μL of each SQ-RT-PCR product was electrophoresed on a 2.0% agarose gel and stained with ethidium bromide.

### Descriptive statistics and exploited bioinformatical tools

For the statistical evaluation of the results, the mean was taken as the measurement of the main tendency, while standard deviation was taken as the dispersion measurement. Differences between groups were analyzed using paired *t*-test and ANOVA. Unless noted otherwise, the threshold for significance was *p* < 0.05. For analyses Software Statistica 12 (StatSoft, Tulsa, OK, USA) was employed. The annotation analyses were performed using the GoMiner (http://discover.nci.nih.gov/gominer/index.jsp), interactome network was constructed using the STRING software (http://string-db.org/) and the PCa metabolic pathway was visualized using Kyoto Encyclopedia of Genes and Genomes (KEGG) pathway database (http://www.genome.jp/kegg/), which provides gold standard sets of molecular pathways. The involvement of genes involved in a cell cycle was carried out using the Reactome (www.reactome.org).

## Results

### Effect of sarcosine on PC-3 cells viability and proliferation *in vitro*

In the first step, we considered pivotal to determine the sarcosine effects on the PC-3 and LNCaP cells viability *in vitro*. Fig 1Aa illustrates that even the lowest applied sarcosine supplementation stimulated the growth of PC-3 cells after 24 h. Noteworthy, the plateau of the stimulation effects was reached using approx. 0.2 μM sarcosine and higher concentrations resulted in slow decreasing viability trends. Similarly, sarcosine treatment stimulated the proliferation of LNCaP cells, but the stimulatory effects were significantly lower than those found in PC-3 cells (Fig 1Ab). As there were obvious impacts on a growth rate of cells, we further analyzed sarcosine influence on their confluency. Light microscopy photographs in Fig 1Ba and 1Bb show that sarcosine supplementation stimulates the proliferation of both PC-3 and LNCaP cells, which can be observed as the increased density of these cells after 72 h cultivation. The found *in vitro* data led us to further proceed to *in vivo* experiments utilizing murine PC-3 and LNCaP xenografts focusing on the effects of sarcosine treatment on a tumor growth and gene expression profiles related to repeated sarcosine supplementation.

**Fig 1:** *In vitro* supplementation of PCa cells with sarcosine. (**A**) Viability (MTT) assay showing the trend in (**Aa**) PC-3 and (**Ab**) LNCaP cells growth under 24 h supplementation with sarcosine (0–10 μM). Values are expressed as the means ± standard deviations of six independent replicates (*n* = 6). (**B**) Micrographs of densities of (**Ba**) PC-3 cultivated in standard Ham’s F12 medium (*left*) and in Ham’s F12 medium enriched for 1 μM sarcosine (*right*) and (**Bb**) LNCaP cultivated in RPMI-1640 medium (*left*) and in RPMI-1640 medium enriched for 1 μM sarcosine (*right*). The length of scale bar is 500 μm.

### Sarcosine treatment effects on growth of tumors *in vivo*

Murine xenografts were induced by using *s*.*c*. inoculation of PCa cells. The experimental workflow of the *in vivo* experiment, showing the treatment course, termination and subsequent analyses is depicted in **Fig 2A**. The results obtained by weighing the treated and non-treated mice demonstrate that in both cases, sarcosine induced significant losses of weight when compared to non-treated individuals [*p* < 0.05, (Fig 2B)]. No mice died or had to be euthanized before the endpoint of the experiment. After the termination, considerable differences between the sizes of excised ectopic prostate tumors were found (Fig 2C), as well as the significant differences in the tumor weights [175 mg *vs*. 94 mg for PC-3 and 137 mg *vs*. 90 mg for LNCaP, *p* < 0.05 (Fig 2D)]. The histological examination of tumor sections however did not reveal any changes within them (Fig 2E).

**Fig 2:** The murine PC-3 and LNCaP xenografts were treated with sarcosine *i*.*p*. (**A**) Schematic depiction of experimental workflow beginning with the PCa cells (5×10^6^) *s*.*c*. inoculation. (**B**) Average weight of mice determined after the termination of experiment. (**C**) Selected photographs of excised ectopic prostate tumors treated with sarcosine (*left*) and non-treated after termination of the experiment (*right*). (**D**) Average tumor weight at the endpoint of the experiment. Values are expressed as the means ± standard deviations of three independent replicates (*n* = 3). Vertical bars indicate standard error. Asterisks indicate significant differences (*p* < 0.05) compared to the untreated group. (**E**) H&E-stained tissue sections of ectopic prostate tumors after treatment with sarcosine (*left*) and non-treated (*right*). The length of scale bar is 100 μm.

### Sarcosine treatment effect on concentration of sarcosine pathway-related amino acids in tumors

As sarcosine pathway involves amino acids providing the essential precursors for the synthesis of proteins, lipids and nucleic acids (particularly serine and glycine), we tested the influence of sarcosine treatment on their tumor tissue concentrations. We also included dimethylglycine (Dmg), the amino acid that can be demethylated by dimethylglycine dehydrogenase to form sarcosine (schematic depiction is shown in Fig 3A). The results found indicate that in PC-3 xenografts, sarcosine treatment resulted in significant (*p* < 0.05) increase in glycine and serine levels (Fig 3B). Moreover, we also detected increased concentrations of sarcosine (0.65 nmol of sarcosine per mg of treated tumor tissue *vs*. 0.43 nmol of sarcosine per mg of non-treated tumor) there. On the other hand, the amount of Dmg was not significantly affected by the sarcosine treatment.

**Fig 3:** Effect of sarcosine treatment on the tumor tissue concentrations of sarcosine pathway-related amino acids. (**A**) Schematic depiction showing the sarcosine pathway ongoing in mitochondrion. Red rectangles highlight the amino acids, whose tissue levels were increased due to sarcosine treatment. Dmg-Dimethylglycine, Gly-Glycine, Ser-Serine, DMGHD-Dimethylglycine dehydrogenase, SARDH-Sarcosine dehydrogenase, GNMT-Glycine-*N*-methyltransferase, GDC-Glycine decarboxylase, SHMT-Serine hydroxymethyltransferase, THF-Tetrahydrofolate, 10f-THF-10-Formyltetrahydrofolate, CH_2_-THF-Methylenetetrahydro-folate, FDH-Formyltetrahydrofolate dehydrogenase, FTS-Formyltetrahydrofolate synthase. Bar graphs showing the differences in tumor tissue Sar, Gly, Dmg and Ser levels in sarcosine treated and non-treated (**B**) PC-3 and (**C**) LNCaP mice. The levels of GNMT and SARDH were estimated in (**D**) PC-3 and (**E**) LNCaP mice by ELISA. Values are means ± standard deviations of three independent replicates (*n* = 3). Asterisks indicate significant differences (*, *p* < 0.05) or (**, *p* < 0.01) compared to the untreated group.

Moreover, Fig 3C demonstrates that LNCaP tumors exhibited very similar response to the sarcosine treatment, having lower initial and induced concentration of sarcosine (0.33 nmol of sarcosine per mg of treated tumor tissue *vs*. 0.19 nmol of sarcosine per mg of non-treated tumor). As GNMT and SARDH are the major enzymes involved in sarcosine metabolism, we further analyzed their amounts within the tumor tissue. Fig 3C and 3D show that sarcosine treatment resulted in significant (*p* < 0.05) increase in concentration of SARDH, which catalyzes sarcosine-to-glycine conversion. In case of GNMT we identified only negligible effects on its amount after sarcosine treatment in both tumor tissues.

### Sarcosine effects on gene expression profiling in tumors

The tumors were further used for isolation of RNA, subsequent reverse transcription and electrochemical microarray profiling (representative microarray heatmaps for the treated and non-treated PC-3 and LNCaP tumors are shown in S1 Fig. Table 1 and Table 2 show the lists of genes (*n* = 43 for PC-3 and *n* = 50 for LNCaP), along with their accession numbers, which were found up-regulated in six independent analyses (*n* = 6). As a threshold for up-regulation, medians, whose fold ratio was ≥ 1.5 compared to non-treated xenografts were exploited. Microarray analyses revealed also seven genes in PC-3 and four genes in LNCaP tumors, which could be classified as down-regulated; however, in both types of cells, none of them reached threshold expression ≤ 1.5 (S1 Table). Thus, they were not considered for further analyses. The complete list of up-regulated genes served as input for further bioinformatical analyses.

**Table 1:** List of genes up-regulated in PC-3 xenografts in a response to sarcosine treatment (genes with the median fold ratio ≥ 1.5 are shown).

Accession No.	Gene name	Symbol	Fold ratio	*p-*value
NM_001071	Thymidylate synthetase	*TYMS*	4.2	0.0016
NM_001323304	Aurora kinase A	*AURKA*	3.7	0.0041
NM_006101	Kinetochore associated 2	*KNTC2*	3.5	0.0012
NM_053056	Cyclin D1	*CCND1*	3.4	0.0004
NM_006469	Influenza virus NS1A binding protein	*IVNS1ABP*	3.1	0.0023
NM_001278547	Mitogen-activated protein kinase 8	*MAPK8*	3.0	0.0067
NM_001302961	Kallikrein 4	*KLK4*	3.0	0.0066
NM_001315	Mitogen-activated protein kinase 14	*MAPK14*	2.6	0.0011
NM_000044	Androgen receptor	*AR*	2.6	0.0024
NM_001030047	Prostate-specific antigen	*KLK3*	2.5	0.0090
NM_001256339	Homeobox protein NK-3 homology A	*NKX3-1*	2.2	0.0016
NM_001281741	Ubiquitin-conjugating enzyme E2C	*UBE2C*	2.2	0.0000
NM_012094	Peroxiredoxin 5	*PRDX5*	2.2	0.0015
NM_001276464	Nuclear receptor subfamily 5, group A	*NR5A2*	2.0	0.0068
NM_001179425	Ribophorin II	*RPN2*	2.0	0.0097
NM_003681	Pyridoxal kinase	*PDXK*	1.9	0.0087
NM_001005915	V-erb-b2 viral oncogene	*ERBB3*	1.9	0.0020
NM_015286	Synemin	*SYNM*	1.9	0.0009
NM_002228	Jun proto-oncogene	*JUN*	1.9	0.0082
NM_001012505	Forkhead box P1	*FOXP1*	1.8	0.0036
NM_001137559	Anaphase promoting complex subunit 5	*ANAPC5*	1.8	0.0030
NM_001291715	Preferentially expressed antigen in melanoma	*PRAME*	1.8	0.0005
NM_006571	Cyclin-dependent kinase inhibitor 1B	*p27*	1.8	0.0012
NM_175620	Metallothionein M	*MTM*	1.7	0.0003
NM_001199149	Lactotransferrin	*LTF*	1.7	0.0012
NM_005494	DnaJ homology, subfamily B, member 6	*DNAJB6*	1.7	0.0082
NM_001077500	Kallikrein 10	*KLK10*	1.7	0.0085
NM_000918	Procollagen-proline, 2-oxoglutarate 4-dioxygenase	*P4HB*	1.7	0.0075
NM_001007226	Speckle-type POZ protein	*SPOP*	1.7	0.0003
NM_001098209	T-cell factor/lymphoid enhancer factor	*TCF/LEF*	1.7	0.0062
NM_000314	Phosphatase and tensin homolog	*PTEN*	1.7	0.0027
NM_002675	Promyelocytic leukemia	*PML*	1.7	0.0023
NM_001291309	Proprotein convertase subtilisin/kexin type 6	*PCSK6*	1.7	0.0033
NM_003183	ADAM metallopeptidase domain 17	*ADAM17*	1.7	0.0003
NM_006191	Proliferation-associated 2G4	*PA2G4*	1.7	0.0005
NM_005066	Splicing factor proline/glutamine-rich	*SFPQ*	1.6	0.0048
NM_001291428	Bcl2-associated X protein	*BAX*	1.6	0.0081
NM_002965	S100 calcium-binding protein A9	*S100A9*	1.6	0.0009
NM_001300960	Cyclin-dependent kinase 19	*CDK19*	1.6	0.0044
NM_006763	BTG family member 2	*BTG2*	1.5	0.0066
NM_006275	Serine/arginine-rich splicing factor 6	*SRSF6*	1.5	0.0023
NM_007203	Paralemmin 2	*PALM2*	1.5	0.0041
NM_001134851	Transcription factor 7	*TCF7*	1.5	0.0025

**Table 2:** List of genes up-regulated in LNCaP xenografts in a response to sarcosine treatment (genes with the median fold ratio ≥ 1.5 are shown).

Accession No.	Gene name	Symbol	Fold ratio	*p*-value
NM_003981	Reticulocalbin 1	*RCN1*	10.0	0.0071
NM_002901	Nuclear receptor subfamily 4, group A, member 3	*NR4A3*	6.6	0.0005
NM_000044	Androgen receptor	*AR*	6.1	0.0001
NM_022002	Breast cancer 1, early onset	*BRCA1*	5.5	0.0069
NM_006191	Proliferation-associated 2G4	*PA2G4*	4.7	0.0042
NM_006571	Cyclin-dependent kinase inhibitor 1B	*p27*	4.1	0.0060
NM_003724	Programmed cell death 2	*PDCD2*	3.9	0.0003
NM_000295	SRY (sex determining region Y)-box 2	*SOX2*	3.7	0.0001
NM_001291715	Preferentially expressed antigen in melanoma	*PRAME*	3.7	0.0087
NM_005033	Procollagen-proline, 2-oxoglutarate 4-dioxygenase	*P4HB*	3.3	0.0036
NM_001302961	Kallikrein 4	*KLK4*	3.1	0.0001
NM_001005915	V-erb-b2 viral oncogene	*ERBB3*	3.1	0.0095
NM_012142	X-box binding protein 1	*XBP1*	2.5	0.0037
NM_005494	DnaJ homology, subfamily B, member 6	*DNAJB6*	2.4	0.0005
NM_004911	Proliferating cell nuclear antigen	*PCNA*	2.4	0.0025
NM_006516	Nuclear factor of kappa light gene inhibitor	*NFKBIA*	2.4	0.0004
NM_001256339	Homeobox protein NK-3 homology A	*NKX3-1*	2.4	0.0063
NM_001005909	B-cell lymphoma 6	*BCL6*	2.3	0.0011
NM_001071	Thymidylate synthetase	*TYMS*	2.3	0.0007
NM_002598	SRY (sex determining region Y)-box 4	*SOX4*	2.3	0.0040
NM_016221	Interleukin 6 (interferon, beta 2)	*IL6*	2.3	0.0000
NM_015927	Nuclear receptor subfamily 4, group A, member 3	*NR4A3*	2.3	0.0033
NM_000314	Phosphatase and tensin homolog	*PTEN*	2.3	0.0014
NM_173158	E2F transcription factor 4	*E2F4*	2.2	0.0040
NM_138320	Asparagine synthetase	*ASNS*	2.2	0.0010
NM_001098209	T-cell factor/lymphoid enhancer factor	*TCF/LEF*	2.1	0.0030
NM_006852	Ubiquitin-conjugating enzyme E2C	*UBE2C*	2.0	0.0036
NM_001137559	Anaphase promoting complex subunit 5	*ANAPC5*	2.0	0.0027
NM_182790	BCL2-associated X protein	*BAX*	2.0	0.0044
NM_000434	Primase, polypeptide 2A	*PRIM2A*	2.0	0.0009
NM_002916	Cathepsin C	*CTSC*	1.9	0.0090
NM_000158	Mitogen-activated protein kinase 7	*MAPK7*	1.9	0.0082
NM_012296	Transforming growth factor, beta 3	*TGFB3*	1.9	0.0010
NM_001030047	Prostate-specific antigen	*KLK3*	1.8	0.0022
NM_015286	Synemin	*SYNM*	1.8	0.0011
NM_015286	Kallikrein 10	*KLK10*	1.8	0.0024
NM_001122	Mitogen-activated protein kinase 10	*MAPK10*	1.8	0.0081
NM_006681	Growth arrest-specific 6	*GAS6*	1.8	0.0006
NM_001001567	ADAM metallopeptidase domain 17	*ADAM17*	1.8	0.0009
NM_007106	Cyclin D2	*CCND2*	1.7	0.0020
NM_004528	BCL2-related protein A1	*BCL2A1*	1.7	0.0071
NM_001470	Splicing factor proline/glutamine-rich	*SFPQ*	1.7	0.0087
NM_138609	Cas-Br-M ecotropic retroviral sequence	*CBL*	1.6	0.0097
NM_004290	Protein kinase, cAMP dependent	*PRKACB*	1.6	0.0067
NM_022805	TIMP metallopeptidase inhibitor 1	*TIMP1*	1.6	0.0015
NM_016237	Replication factor C	*RFC4*	1.6	0.0087
NM_020738	Protein kinase C, beta 1	*PRKCB1*	1.5	0.0068
NM_000593	Transcription factor 7 (T-cell specific, HMG-box)	*TCF7*	1.5	0.0011
NM_003290	Integrin, beta 5	*ITGB5*	1.5	0.0039
NM_014573	Proteasome (prosome, macropain) subunit	*PSMD2*	1.5	0.0098

### SQ-RT-PCR validation of microarray data

Overall, our microarray analyses revealed 18 overlapping genes, which were up-regulated in both tested PCa cell lines as the response to sarcosine treatment (Fig 4A). To validate the microarray results, we performed SQ-RT-PCR analyses using the sarcosine treated and non-treated tumors and evaluated gene expression after normalization according to the expression of *β-actin*. Fig 4B shows the SQ-RT-PCR results for the most up-regulated genes, which were selected for validation (up-regulation fold ratio ≥ 2.5). Noteworthy, all of the results corroborated our microarray analyses and confirmed the considerable influence on genes expression caused by sarcosine administration.

**Fig 4:** Comparison of gene expression in PC-3 and LNCaP xenografts. (**A**) Venn diagram showing the number of overlapping genes up-regulated after treatment of PC-3 and LNCaP cells with sarcosine. (**B**) SQ-RT-PCR validation of 10 selected genes up-regulated in murine PC-3 and LNCaP xenografts after sarcosine treatment (up-regulation ≥ 2.5). Expression of *β-actin* constituted as loading control. Lanes **1**–**3**—RNA isolated from sarcosine treated mice, lane **4**–**6**—RNA isolated from non-treated mice.

### Classification of biological roles of genes influenced by sarcosine treatment

To evaluate biological relevance of the differentially expressed genes in sarcosine treated and non-treated prostate tumors, we carried out an annotation analysis, which identifies the involvement of particular genes within biological processes. For both types of PCa cells xenografts, the up-regulated gene set was found to mostly include the genes belonging to "metabolic process", "cellular process", "biological regulation", "response to stimulus", "developmental process", "apoptotic process" and others (Table 3). Taken together this analysis provided a preliminary insight into the function of genes that are up-regulated as a response to sarcosine treatment.

**Table 3:** Percentage of genes up-regulated in ectopic prostate xenografts treated with sarcosine classified with respect to their biological functions.

	PC-3	LNCaP
Gene biological process	% of total genes	% of total genes
Metabolic process	55.8	52.0
Cellular process	44.2	51.5
Biological regulation	26.7	36.5
Response to stimulus	20.0	15.5
Developmental process	20.0	14.8
Apoptotic process	15.8	23.2
Multicellular organism process	10.8	26.1
Cellular component organization or biogenesis	5.8	10.1
Reproduction	5.8	3.1
Immune system process	5.0	4.2
Locomotion	2.5	1.1
Biological adhesion	2.5	2.0

Further, to prioritize the differentially expressed genes involved in the apoptosis and cell cycle, which are the major hallmarks of each type of cancer, we utilized STRING database of known and predicted interactions. Fig 5 illustrates the interactome network, where the red nodes highlight the genes from our up-regulated set, whose expression is stimulated by sarcosine treatment and which may be involved in a cell death of PC-3 cells (namely *FOXP1*, *LTF1*, *TCF7*, *DNAJB6*, *JUN*, *MAPK8*, *ERBB3*, *BTG2*, *AURKA*, *PA2G4*, *PML*, *PRDX5*, *PRAME* and *IVNS1ABP*) and LNCaP cells (namely *ITGA6*, *BRCA1*, *CBL*, *ERBB3*, *PA2G4*, *KLF4*, *MAPK7*, *ASNS*, *SOX4*, *TCF7*, *NR4A3*, *TGFB3*, *GAS6*, *TIMP1*, *BAX*, *BCL2A1*, *NFKBIA*, *HSP9OB1*, *DNAJB6*, *XBP1*, *BCL6* and *PRAME*). Noteworthy, *TCF7*, *DNAJB6*, *ERBB3* and *PRAME* were up-regulated in both types of cells pointing out their importance for cell cycle and apoptosis of metastatic PCa cells.

**Fig 5:** Interactome network showing the genes, which were up-regulated after sarcosine treatment and which are fundamental for apoptosis and cell cycle (PC-3 on the left, LNCaP on the right). The red nodes highlight the genes, which were up-regulated and are involved in negative regulation of a cell death. The interior of the circle represents the structure of proteins. The color of the line provides evidence of the different interactions among proteins. A red line indicates the presence of fusion evidence; a green line, neighborhood evidence; a blue line, concurrence evidence; a purple line, experimental evidence; a light blue line, database evidence; a black line, coexpression evidence. The genes were analyzed using STRING software (version 10.0).

### Sarcosine and induction of genes involved in PCa-specific metabolic pathway and cell cycle

Further, we analyzed the expression changes associated with the PCa biochemical pathway defined in the KEGG database [17]. It is worth noting that KEGG pathway maps are an abbreviated representation of known interactions, focusing on those considered being the best supported by the evidence and relevance. Fig 6 and Fig 7 show the PCa metabolic pathway-specific KEGG diagrams, where the up-regulated genes are highlighted in red. Noteworthy, these genes are involved in the most fundamental processes, such as the cell proliferation and survival [*TCF/LEF*, *KLK3* (or *PSA*)], cell cycle and its progression (*p27*), PI3K/Akt signaling pathway (*NKX3*.*1* and *PTEN*) and hormone signaling (*AR*). The diagrams underscore that in both metastatic PCa cells, sarcosine affects nearly the same targets involved in fundamental metabolic processes. Fig 8 demonstrates a general cell cycle and the phases of mitosis. This detailed insight into the specific effects of sarcosine treatment revealed that in PC-3 tumors, sarcosine up-regulates genes, which are vital for a cell cycle, such as *RPN2* involved in all cell cycle phases, *UBE2C* involved in S phase and M phase (specifically prometaphase and anaphase), *KNTC2* and *ANAPC5* involved in S and M phases, *TYMS* and *CCND1* involved in G_1_-G_1_/S phases and *SYNM* involved in G_2_-G_2_/M phases. Fig 8 illustrates that similarly, in LNCaP tumors, sarcosine affects a cell cycle. Remarkably, up-regulation of *ANAPC5*, *SYNM* and *UBEC2C* and *TYMS* was identified within both tumor tissues exposed to sarcosine, irrespective of androgen dependence. Overall, the sarcosine-induced up-regulation of cell cycle controlling genes is likely one of the factor standing behind the sarcosine treatment-stimulated PCa cells proliferation and tumor growth.

**Fig 6:** KEGG PCa-specific metabolism diagram for PC-3 cells. Gene expression shifts are projected as comparison of sarcosine treated and non-treated prostate tumors. The genes highlighted in red were found up-regulated after the sarcosine treatment in both PCa xenografts. The pathway map is species-specific (*Homo sapiens*).

**Fig 7:** KEGG PCa-specific metabolism diagram for LNCaP cells. Gene expression shifts are projected as comparison of sarcosine treated and non-treated prostate tumors. The genes highlighted in red were found up-regulated after the sarcosine treatment in both PCa xenografts. The pathway map is species-specific (*Homo sapiens*).

**Fig 8:** Schematic depiction of cell cycle and illustration of genes, which induce progression of cell cycle, performed using the Reactome software. Black frames indicate the genes, which were up-regulated after sarcosine treatment.

## Discussion

PCa remains a leading cause of illness and death among men in the US and Western Europe. The optimal course of treatment for a given individual is often uncertain. Recent metabolomic studies have identified various oncometabolites of PCa that could be likely associated with aggressive disease [2, 18, 19]. However, an understanding the biological actions of these molecules is anticipated to provide valuable information that can be helpful not only for enhancement of diagnostic and prognostic possibilities, but also for the development of novel biological treatment agents.

Numerous studies highlighted the significance of sarcosine as oncometabolite in PCa progression [2–4, 10]. Previously, we showed that sarcosine supplementation stimulates the cell proliferation and decreased the time required for cell division in malignant (22Rv1) and metastatic (PC-3) PCa cells [8]. In the present work we show that sarcosine exhibits considerable stimulatory effects on growth of PC-3 and LNCaP cells, even at very low concentrations, which are comparable to those found in urinary specimens of subjects suffering from aggressive PCa [3]. Similar efforts were put by Khan and coworkers using benign DU145 prostate cells as it was found that sarcosine did not affect their ability to progress through the cell cycle or impair cell proliferation [10]. Thus, these findings, which are in good agreement with ours, highlight the particular importance of sarcosine in malignant/metastatic prostate cells.

Despite that an utilization of *in vivo* preclinical model is critical for complex understanding of the actions triggered by sarcosine treatment, we established a system that mimics the tumor biology and its microenvironment by using xenografts. Sarcosine treatment of PC-3 and LNCaP xenografts resulted in a significant decrease (*p* ˂ 0.05) in weight of treated mice, concomitantly with the increased size of their tumors. This indicates the stimulation of cancer progression with simultaneous deterioration of the conditions of treated animals. Previously, it has been demonstrated that stable overexpression of the SARDH enzyme or knock-down of the GNMT enzyme led to inhibition of the growth of PCa xenografts [10]. Nevertheless, the effect of direct sarcosine supplementation was not investigated. Hence, in this work, we provide further evidence of the stimulatory effects of sarcosine on a model of androgen dependent (LNCaP) and androgen independent (PC-3) metastatic PCa, which was firstly studied on a level of the impact on free amino acids and enzymes, which are involved in sarcosine biosynthesis and/or conversion schematized in Fig 3A.

Moreover, our results revealed sarcosine-induced increase of glycine and serine within the tumor mass formed by both types of PCa cells. In general, cancer cells undergo specific metabolic reprogramming to sustain cell growth and proliferation [20]. In addition to a large energy requirement, they tend to accumulate building blocks for the construction of new cellular components including nucleic acids, proteins, and lipids, as well as important cofactors for the maintenance of the cellular redox status [21]. The importance of serine and glycine as precursors in those processes is comprehensively summarized in the review by Amelio and coworkers [22]. Briefly, both serine and glycine contribute to cellular metabolism through the glycine cleavage system, which refuels one-carbon metabolism based on chemical reactions of folate compounds [23]. The importance of folate metabolism is underlined by the fact that antifolate chemotherapy is currently widely used in cancer treatment [24]. Similarly to serine and glycine, we also identified significantly higher amount of sarcosine, but not its precursor—dimethylglycine. Sarcosine likely accumulates within the tumor mass with the consequent increase in serine and glycine, which act as the tumor growth promoters. As it was evidenced, sarcosine increased amount also stimulates the SARDH expression. Although there is a lack of direct evidence of linkage between SARDH and PCa aggressiveness, Yoon and coworkers demonstrated that the expression of SARDH is associated with shorter overall survival of subjects suffering from luminal A type breast cancer [25]. Although here we report obvious effects of sarcosine treatment on its pathway *in vivo*, further analysis of metabolic activities of sarcosine associated enzymes might be done to shed more light into this phenomenon.

As another level of regulation, we further investigated the differential gene expression sets related to sarcosine treatment. Particularly, we exploited electrochemical DNA microarrays, which are designated to analyze 2000 genes, involved in any aspect of cancer disease. Such approach provides a complex insight into the expression of genes that are involved in regulation of cell cycle and apoptosis, which are the major hallmarks of cancer [11]. Within the set of the identified differentially expressed genes, we found significant up-regulation of genes involved in a regulation of cell cycle and genes stimulating cell proliferation. Interestingly, in both types of PCa cells, we also identified sarcosine-related up-regulation of gene encoding androgen receptor (AR), which is a transcription factor mediating the transcription of both SARDH and GNMT [26].

TYMS enzyme (encoded by *TYMS*) plays a role in DNA synthesis and G_1_-S transition. Its expression is higher in neoplastic than in normal prostate epithelium and was shown to be tightly linked to high GS, pathological tumor stage and early PSA recurrence (*p* < 0.0001) [27]. Noteworthy, TYMS protein is important target for 5-fluorouracil (5-FU) treatment, however this drug has only limited response rates in PCa [28]. Our findings encourage further studies to compare the expression of TYMS and amounts of urinary sarcosine, which can be exploited as non-invasive predictor of success of 5-FU chemotherapy.

Similarly, *AURKA* gene amplification has been documented in 67% of neuroendocrine PCa, which progress to highly aggressive variants [29]. *CCND1* overexpression accounts for cisplatin resistance through cell cycle control and inhibits cellular apoptosis pathway in the most of tumors [30]. Overexpression of *KLK4* was observed in patients with high T stage and GS [31] and *KLK3* encodes PSA, a widely used biomarker for PCa detection and disease monitoring [32]. *KNTC2* encodes the Hec1 protein, which plays an essential role in chromosome segregation by interacting through its coiled-coil domains with several proteins modulating the G_2_/M transition [33]. Hec1 is a critical modulator of mitosis, highly expressed in most cancer cells, including PCa [34], however in this case the comparison of their expression with sarcosine amounts was not carried out, too.

In LNCaP tumors, we found that the most up-regulated gene was *RCN1*; encoding the homonymous protein RCN1, which has been identified as surface adhesion molecule that might participate in metastasis of PCa [35]. *NR4A3* is a member of the orphan nuclear receptor family referred to as NR4A. These receptors have been implicated in cell cycle regulation, apoptosis and carcinogenesis [36]. As it has been found that *NR4A3* controls both, survival and cell death of cancer cells, it is worth noting that sarcosine significantly stimulates its up-regulation, which can be one of the mechanisms of PCa proliferation.

In both types of PCa xenografts, we have revealed that sarcosine treatment stimulated the expression of AR, whose activity was intimately linked to PCa. Kim *et al*. show that AR and sarcosine metabolism-related enzymes have significant relationships with each other [37] and androgens can increase GNMT expression through AR binding the androgen response element existing on the first exon coding region of *GNMT*. Similarly, Sreekumar and coworkers indicated that AR appears to directly regulate sarcosine levels *via* transcriptional control of its regulatory enzymes [2]. Nevertheless, the principle of the *vice versa* mechanism (sarcosine stimulation of AR expression) needs to be clarified. Recently, it was demonstrated that exogenous addition of sarcosine to LNCaP cells *in vitro* caused negligible stimulation of AR expression only [38]. Discrepancy in our results is likely due to the experimental level (*in vitro vs*. *in vivo*), where the induced tumors can be influenced by hormones floating in the bloodstream of the host organism. Overall, we anticipate that the linkage between androgen signaling and sarcosine metabolism may be vital for a development and progression of PCa and further research on this phenomenon may provide valuable information into the biology of these malicious diseases.

On the other hand, in PC-3 tumors, we have identified sarcosine-related up-regulation of *MAPK8* and *MAPK14*, which act as integration points for multiple biochemical signals and affect cellular processes, including proliferation [39]. Both *MAPK8* (encoding JNK1) and MAPK14 (encoding p38) signaling pathways are activated by pro- or anti-inflammatory cytokines, but also in response to cellular stress (genotoxic, osmotic, hypoxic or oxidative) to cause growth inhibition and apoptosis [40]. Contrary to that, it was also demonstrated that both JNK1 and p38 can act as PCa promoters. This depends on the cell type and specific stimuli inducing the ability to regulate cell adhesion, invasion and migration [41]. Considering all found results, it is obvious that sarcosine treatment did not exert significant antitumor action through up-regulation of *MAPK8* and *MAPK14*. Similar phenomenon has been identified in case of *p27* as the cyclin-dependent kinase inhibitor regulating cell proliferation, motility and apoptosis. Interestingly, it can exert both a positive and a negative action on these processes in dependence on diverse post-translation modifications [42]. We did not find any expression in non-treated LNCaP tumors; however sarcosine exposure resulted in a significant up-regulation of *p27*. Further studies on a protein level might be performed to investigate, whether the gene expression correlates with the protein amount and to elucidate, whether the protein translated in response to sarcosine presence, behaves as the good or the bad one. Overall, we show that sarcosine plays a pivotal role in influencing metastatic PCa cells, irrespective of androgen dependence status.

## Conclusion

The present study demonstrates that sarcosine treatment stimulates the PCa cells, both *in vitro* and *in vivo*. Our results indicate that direct, repeated administration to sarcosine has significant stimulatory effects on the growth of ectopic prostate tumors. Further biochemical and molecular-biology analyses revealed considerable impact of treatment on sarcosine metabolic pathway and the expression of genes involved in cell proliferation, cell cycle and apoptosis, which are the major hallmarks of each cancer. To the best of our knowledge, this is the first study showing the direct effects of repeated sarcosine treatment on an organism bearing prostate tumor. Despite the complexity of obtained data, there are still questions arising, including the impact of enzymatic activities of sarcosine metabolism enzymes on PCa development. Moreover, our results might be verified by a detailed proteomic screening. Despite those facts, the present study confirmed sarcosine as important PCa oncometabolite in both androgen dependent and androgen independent metastatic PCa cells, and provided pivotal information, which could be further investigated and developed.

## Supporting Information

S1 Fig ElectraSense microarray heatmaps, where each spot represents expression of one gene (gray scale intensity describes the rate of individual mRNA expression). (DOCX)

S1 Table List of genes down-regulated in PC-3 and LNCaP xenografts in a response to sarcosine treatment. (DOCX)

## References

[1] CerneiN, HegerZ, GumulecJ, ZitkaO, MasarikM, BabulaP, et al Sarcosine as a Potential Prostate Cancer Biomarker-A Review. Int J Mol Sci. 2013;14(7):13893–908. 10.3390/ijms140713893 .23880848PMC3742224

[2] SreekumarA, PoissonLM, RajendiranTM, KhanAP, CaoQ, YuJD, et al Metabolomic profiles delineate potential role for sarcosine in prostate cancer progression. Nature. 2009;457(7231):910–4. 10.1038/nature07762 .19212411PMC2724746

[3] HegerZ, CerneiN, GumulecJ, MasarikM, EckschlagerT, HrabecR, et al Determination of common urine substances as an assay for improving prostate carcinoma diagnostics. Oncol Rep. 2014;31(4):1846–54. 10.3892/or.2014.3054 .24573566

[4] KumarD, GuptaA, MandhaniA, SankhwarSN. Metabolomics-Derived Prostate Cancer Biomarkers: Fact or Fiction? J Proteome Res. 2015;14(3):1455–64. 10.1021/pr5011108 .25609016

[5] HegerZ, CerneiN, KrizkovaS, MasarikM, KopelP, HodekP, et al Paramagnetic Nanoparticles as a Platform for FRET-Based Sarcosine Picomolar Detection. Sci Rep. 2015;5:1–7. 8868 10.1038/srep08868 .PMC435285925746688

[6] AnkerstDP, LissM, ZapataD, HoeflerJ, ThompsonIM, LeachRJ. A case control study of sarcosine as an early prostate cancer detection biomarker. BMC Urol. 2015;15:1–4. 99 10.1186/s12894-015-0095-5 .PMC459162826429735

[7] JentzmikF, StephanC, MillerK, SchraderM, ErbersdoblerA, KristiansenG, et al Sarcosine in Urine after Digital Rectal Examination Fails as a Marker in Prostate Cancer Detection and Identification of Aggressive Tumours. Eur Urol. 2010;58(1):12–8. 10.1016/j.eururo.2010.01.035 .20117878

[8] HegerZ, GumulecJ, CerneiN, PolanskaH, RaudenskaM, MasarikM, et al Relation of exposure to amino acids involved in sarcosine metabolic pathway on behavior of non-tumor and malignant prostatic cell lines. Prostate. 2016;76(7):679–90. 10.1002/pros.23159 .26847870

[9] SudhakaranPR, BinuS, SoumyaSJ. Effect of sarcosine on endothelial function relevant to angiogenesis. J Canc Res Ther. 2014;10(3):603–10. 10.4103/0973-1482.137945 .25313747

[10] KhanAP, RajendiranTM, AteeqB, AsanganiIA, AthanikarJN, YocumAK, et al The Role of Sarcosine Metabolism in Prostate Cancer Progression. Neoplasia. 2013;15(5):491–501. 10.1593/neo.13314 .23633921PMC3638352

[11] EvanGI, VousdenKH. Proliferation, cell cycle and apoptosis in cancer. Nature. 2001;411(6835):342–8. 10.1038/35077213 .11357141

[12] GeschwindDH. DNA microarrays: translation of the genome from laboratory to clinic. Lancet Neurol. 2003;2(5):275–82. 10.1016/s1474-4422(03)00379-x .12849181

[13] LipshutzRJ, FodorSPA, GingerasTR, LockhartDJ. High density synthetic oligonucleotide arrays. Nature Genet. 1999;21:20–4. 10.1038/4447 .9915496

[14] HegerZ, CerneiN, KudrJ, GumulecJ, BlazkovaI, ZitkaO, et al A Novel Insight into the Cardiotoxicity of Antineoplastic Drug Doxorubicin. Int J Mol Sci. 2013;14(11):21629–46. 10.3390/ijms141121629 .24185911PMC3856025

[15] RothKM, PeyvanK, SchwarzkopfKR, GhindilisA. Electrochemical detection of short DNA oligomer hybridization using the CombiMatrix ElectraSense Microarray reader. Electroanalysis. 2006;18(19–20):1982–8. 10.1002/elan.200603603 .

[16] HegerZ, MichalekP, GuranR, HavelkovaB, KominkovaM, CerneiN, et al Exposure to 17 beta-Oestradiol Induces Oxidative Stress in the Non-Oestrogen Receptor Invertebrate Species Eisenia fetida. PLoS One. 2015;10(12). e0145426 10.1371/journal.pone.0145426 .PMC469059326695684

[17] KanehisaM, GotoS, FurumichiM, TanabeM, HirakawaM. KEGG for representation and analysis of molecular networks involving diseases and drugs. Nucleic Acids Res. 2010;38:D355–D60. 10.1093/nar/gkp896 .19880382PMC2808910

[18] DingZH, WuCJ, ChuGC, XiaoYH, HoD, ZhangJF, et al SMAD4-dependent barrier constrains prostate cancer growth and metastatic progression. Nature. 2011;470(7333):269–73. 10.1038/nature09677 .21289624PMC3753179

[19] TomlinsSA, AubinSMJ, SiddiquiJ, LonigroRJ, Sefton-MillerL, MiickS, et al Urine TMPRSS2:ERG Fusion Transcript Stratifies Prostate Cancer Risk in Men with Elevated Serum PSA. Sci Transl Med. 2011;3(94). 94ra72 10.1126/scitranslmed.3001970 .PMC324571321813756

[20] HeidenMGV, CantleyLC, ThompsonCB. Understanding the Warburg Effect: The Metabolic Requirements of Cell Proliferation. Science. 2009;324(5930):1029–33. 10.1126/science.1160809 .19460998PMC2849637

[21] LocasaleJW. Serine, glycine and one-carbon units: cancer metabolism in full circle. Nat Rev Cancer. 2013;13(8):572–83. 10.1038/nrc3557 .23822983PMC3806315

[22] AmelioI, CutruzzolaF, AntonovA, AgostiniM, MelinoG. Serine and glycine metabolism in cancer. Trends BiochemSci. 2014;39(4):191–8. 10.1016/j.tibs.2014.02.004 .PMC398998824657017

[23] BrosnanME, MacMillanL, StevensJR, BrosnanJT. Division of labour: how does folate metabolism partition between one-carbon metabolism and amino acid oxidation? Biochem J. 2015;472:135–46. 10.1042/bj20150837 .26567272

[24] MarchettiC, PalaiaI, GiorginiM, De MediciC, IadarolaR, VertechyL, et al Targeted drug delivery via folate receptors in recurrent ovarian cancer: a review. OncoTargets Ther. 2014;7:1223–36. 10.2147/ott.s40947 .PMC409649125031539

[25] YoonJK, KimDH, KooJS. Implications of differences in expression of sarcosine metabolism-related proteins according to the molecular subtype of breast cancer. J Transl Med. 2014;12 149 10.1186/1479-5876-12-149 .PMC404590424884785

[26] GreenT, ChenXF, RyanS, AschAS, Ruiz-EchevarriaMJ. TMEFF2 and SARDH cooperate to modulate one-carbon metabolism and invasion of prostate cancer cells. Prostate. 2013;73(14):1561–75. 10.1002/pros.22706 .23824605PMC3878307

[27] BurdelskiC, StraussC, TsourlakisMC, KluthM, Hube-MaggC, MellingN, et al Overexpression of thymidylate synthase (TYMS) is associated with aggressive tumor features and early PSA recurrence in prostate cancer. Oncotarget. 2015;6(10):8377–87. 10.18632/oncotarget.310725762627PMC4480759

[28] BrodyJR, HuclT, CostantinoCL, EshlemanJR, GallmeierE, ZhuH, et al Limits to Thymidylate Synthase and TP53 Genes as Predictive Determinants for Fluoropyrimidine Sensitivity and Further Evidence for RNA-Based Toxicity as a Major Influence. Cancer Res. 2009;69(3):984–91. 10.1158/0008-5472.can-08-3610 .19155291PMC2887094

[29] ParkK, ChenZM, MacDonaldTY, SiddiquiJ, YeHH, ErbersdoblerA, et al Prostate cancer with Paneth cell-like neuroendocrine differentiation has recognizable histomorphology and harbors AURKA gene amplification. Hum Pathol. 2014;45(10):2136–43. 10.1016/j.humpath.2014.06.008 .25128228PMC4414025

[30] ZhouXJ, ZhangZY, YangX, ChenWT, ZhangP. Inhibition of cyclin D1 expression by cyclin D1 shRNAs in human oral squamous cell carcinoma cells is associated with increased cisplatin chemosensitivity. Int J Cancer. 2009;124(2):483–9. 10.1002/ijc.23964 .18942709

[31] MukaiS, YoritaK, YamasakiK, NagaiT, KamibeppuT, SugieS, et al Expression of human kallikrein 1-related peptidase 4 (KLK4) and MET phosphorylation in prostate cancer tissue: immunohistochemical analysis. Hum Cell. 2015;28(3):133–42. 10.1007/s13577-015-0114-6 .25862631

[32] Kote-JaraiZ, Al OlamaAA, LeongamornlertD, TymrakiewiczM, SaundersE, GuyM, et al Identification of a novel prostate cancer susceptibility variant in the KLK3 gene transcript. Hum Genet. 2011;129(6):687–94. 10.1007/s00439-011-0981-1 .21465221PMC3092928

[33] WangHF, GaoX, LuX, WangY, MaCF, ShiZK, et al The mitotic regulator Hec1 is a critical modulator of prostate cancer through the long non-coding RNA BX647187 in vitro. Biosci Rep. 2015;35 e00273 10.1042/bsr20150003 .PMC466058126612002

[34] ChenYM, RileyDJ, ZhengL, ChenPL, LeeWH. Phosphorylation of the mitotic regulator protein Hec1 by Nek2 kinase is essential for faithful chromosome segregation. J Biol Chem. 2002;277(51):49408–16. 10.1074/jbc.M207069200 .12386167

[35] CooperCR, GravesB, PruittF, ChaibH, LynchJE, CoxAK, et al Novel surface expression of reticulocalbin 1 on bone endothelial cells and human prostate cancer cells is regulated by TNF-alpha. J Cell Biochem. 2008;104(6):2298–309. 10.1002/jcb.21785 .18561328

[36] DeutschAJA, AngererH, FuchsTE, NeumeisterP. The Nuclear Orphan Receptors NR4A as Therapeutic Target in Cancer Therapy. Anti-Cancer Agents Med Chem. 2012;12(9):1001–14. .10.2174/18715201280352961922583411

[37] KimMJ, JungWH, KooJS. Expression of sarcosine metabolism-related proteins in estrogen receptor negative breast cancer according to the androgen receptor and HER-2 status. Int J Clin Exp Pathol. 2015;8(7):7967–77. .26339363PMC4555691

[38] DahlM, BoucheloucheP, Kramer-MarekG, CapalaJ, NordlingJ, BoucheloucheK. Sarcosine induces increase in HER2/neu expression in androgen-dependent prostate cancer cells. Mol Biol Rep. 2011;38(7):4237–43. 10.1007/s11033-010-0442-2 .21755295PMC3402037

[39] TiwariN, Meyer-SchallerN, ArnoldP, AntoniadisH, PachkovM, van NimwegenE, et al Klf4 Is a Transcriptional Regulator of Genes Critical for EMT, Including Jnk1 (Mapk8). PLoS One. 2013;8(2). e57329 10.1371/journal.pone.0057329 .PMC358148923451207

[40] JunttilaMR, LiSP, WestermarckJ. Phosphatase-mediated crosstalk between MAPK signalling pathways in the regulation of cell survival. Faseb J. 2008;22(4):954–65. 10.1096/fj.06-7859rev .18039929

[41] ChienCS, ShenKH, HuangJS, KoSC, ShihYW. Antimetastatic potential of fisetin involves inactivation of the PI3K/Akt and JNK signaling pathways with downregulation of MMP-2/9 expressions in prostate cancer PC-3 cells. Mol Cell Biochem. 2010;333(1–2):169–80. 10.1007/s11010-009-0217-z .19633975

[42] ChuIM, HengstL, SlingerlandJM. The Cdk inhibitor p27 in human cancer: prognostic potential and relevance to anticancer therapy. Nat Rev Cancer. 2008;8(4):253–67. 10.1038/nrc2347 .18354415

